# A Stock Selection Model of Image Classification Method Based on Convolutional Neural Network

**DOI:** 10.1155/2022/4743427

**Published:** 2022-05-20

**Authors:** Pengfei Li, Jungang Xu, Keyao Li

**Affiliations:** University of Chinese Academy of Sciences, Beijing, China

## Abstract

With the development of artificial intelligence technology, an increasing number of researchers try to apply different machine learning and deep learning methods to quantitative trading fields to obtain more stable and efficient trading models. As a typical quantitative trading strategy, stock selection has also attracted a lot of attention. There are many studies and applications on stock selection. However, the existing research and application cannot meet the continuous expansion of the scale and dimension of stock selection data set and cannot meet the needs in terms of efficiency and accuracy of stock selection. A convolutional neural network has been applied to image classification and achieved better results than the traditional methods. In this study, we first constructed a multifactor stock selection data set based on China's stock market. Then, we apply the convolutional neural network model to analyze stock selection data and select stocks. The main contribution of this study is that we build a stock multifactor data set, construct a “factor picture,” and classify them by convolutional neural network to select stocks. This study also makes comparative experiments on the decision tree, support vector machine, and feedforward neural network in stock selection on the same data set constructed in this study. The results show that the stock selection method based on the convolutional neural network outperforms other methods in terms of the annual return, sharp ratio, and max drawdown.

## 1. Introduction

At present, China's stock market is becoming larger and larger, the market environment is becoming more and more open, the market situation is more stable, and the market profitability has been greatly improved. The huge development potential of China's stock market has attracted more and more investment institutions and individuals at home and abroad to enter the China's investment market. However, financial investment is an area with relatively small fault tolerance. Especially in the stock market, ordinary investors have a low fault tolerance rate; in other words, a wrong transaction may cause large losses. Most of this loss is irreversible, which leads to a lot of individuals being forced to withdraw from the stock market. The complex and changeable market environment hinders the return and stability of quantitative trading strategy. Therefore, people try to use computer technology to analyze the stock data, hoping to get effective trading rules, build reusable trading strategies, and improve the return and stability of quantitative trading strategy, so as to protect the interests of investors and maintain the stability of financial market.

Quantitative trading is a new way of financial trading. Compared with traditional subjective trading, quantitative trading has the characteristics of system and discipline. It is widely used in the analysis and trading of stocks, futures, bonds, and other financial varieties. According to different strategic logic, quantitative trading can be divided into stock selection, quantitative timing, high-frequency trading, and statistical arbitrage. With the continuous development and integration of different fields, quantitative trading has become the product of the combination of statistics, finance, marketing, economics, and computer science.

As a typical quantitative trading strategy, stock selection refers to the process of establishing a model by using methods to screen listed stocks and obtain income by selecting stocks with better performance in the future [1]. The key of stock selection is to mine the driving factors behind the stock price and then analyze the internal relationship between these factors, so as to find the relationship between the stock price and the stock value and then trade the stocks with profit value. A good stock selection strategy should consider not only its profitability but also its risk control ability, so as to ensure the return and stability of the quantitative stock selection strategy.

From the traditional index analysis method, to the use of statistical methods for stock selection, and then to the current artificial intelligence method represented by machine learning, stock selection has undergone great changes. Machine learning is currently used in many fields, including computer vision [2, 3], image processing [4], natural language processing [5–7], speech recognition [8, 9], etc. In the field of stock selection, machine learning methods are used widely. Stock selection strategy can be divided as follows: analytic hierarchy process [10–12], principal component analysis [13–15], clustering [16–18], evolutionary algorithms [19–21], support vector machine [22–24], artificial neural network [25–27], and random forest [28, 29].

There are many studies using the machine learning method to select stocks. In 2009, Becker [30] provided a stock selection model using genetic programming. The decision variables used in the model are financial factors determined by experts. The experimental results show that the genetic programming method can build a multifactor stock selection model and then sort the stocks in S&P500 to select the high-yield stock portfolio. In 2015, Zikowski [31] proposed a volume-weighted support vector machine (VW-SVM) model to select features through the Fisher method and introduce the delay of technical indicators to expand the training vector, so as to realize short-term stock (portfolio) selection. The experimental results show that the model is better than the traditional SVM model and has a better stock selection income. In 2018, Li [32] constructed a stock selection method combining improved Gaussian kernel function and K-means clustering, which improved the ability of K-means model to deal with high-dimensional and linear inseparable problems through Gaussian function, while the complexity of the algorithm did not change. The experimental results proved that the model can achieve higher stock selection excess return. In 2021, Liu et al. [33] proposed a hybrid model based on grey wolf optimization and support vector regression. Compared with a genetic algorithm, particle swarm optimization and other optimization algorithms, grey wolf optimization improves the prediction performance of support vector regression and can achieve better income and higher stability in China's stock market.

Stock data is one of the financial data with the characteristic of time series. With the continuous growth of data dimension and the continuous expansion of data scale, the existing stock selection methods are difficult to extract effective features from stock data, and the performance and efficiency of stock selection are greatly limited. Although some studies have focused on the study of stock selection factors, there are still some complex problems. The stock selection strategies based on different machine learning methods have achieved good experimental results, but we still find the following two main problems in the field of stock selection:

The first problem is that the feature extraction of high-dimensional data is still a complex work, especially in stock selection. Due to the large dimension and rich types of stock selection factors, it is difficult to select different types of factors, while invalid factors seriously affect the accuracy and efficiency of stock selection model;

The second problem is that traditional machine learning methods are difficult to extract features, and the classification effect is poor. In particular, the stock selection model based on traditional machine learning is easy to be affected by the data set, so it is difficult to obtain a long-term stable and effective stock selection model.

Therefore, we propose the following corresponding solutions in this study to solve the two main problems:

First, by calculating the correlation between stock selection factors and combining the factors with low correlation, we finally realize the feature extraction of stock selection factors and construct a multifactor stock selection data set.

Second, deep learning has inherent advantages in dealing with high-dimensional and large-scale complex data sets. As a typical deep learning method, the convolutional neural network (CNN) can effectively learn the corresponding features from a large number of samples, avoid the complex feature extraction process, and achieve very good results for classification tasks. Therefore, it is widely used in the fields of image classification, target recognition, and speech recognition. Therefore, in order to process and analyze the high-dimensional and large-scale stock data, so as to select the stock portfolio with high return, we propose a stock selection method based on CNN. Taking advantage of CNN's image classification, we realize the stock classification by constructing a “factor picture,” so as to achieve the purpose of stock selection.

Finally, we test the stock selection models of decision tree, support vector machine (SVM), and feedforward neural network (FNN) on the same data set and compare and analyze the results, so as to verify that the multifactor stock selection data set and the stock selection method based on the CNN can increase the return and stability of stock selection.

The rest of the study is structured as follows: in Section 2, we explain the construction process of multifactor stock selection data set.  Section 3 focuses on the construction process of stock selection model based on CNN. In Section 4, the results of the stock selection method based on CNN are shown, and the advantages of the stock selection model based on CNN are obtained by comparing with the methods based on decision tree, SVM, and FNN. Finally, we summarize the stock selection method based on CNN.

## 2. Multifactor Stock Selection Data Set

In order to build a multifactor stock selection data set, we collect data from the data platform named tushare and the website named eastmoney.com. The data types collected include the fundamental data of all listed companies in China's stock market and some technical index data. The data set spans from 2008 to 2020. The fundamental data are mainly from the financial statement data released by listed companies. In China, the financial statement data released mainly include a balance sheet, cash flow statement, and income statement. These three types of statements reflect the company's financial situation in this period. We think the operating conditions reflected in the financial statements will be reflected in the stock price. Therefore, we choose our factors in the three financial statements. In addition, in order to enrich the factors, we also added the technical stock selection factors to the factor set. Finally, we constructed a quantitative stock selection factor set including fundamental factors and technical factors. The dimension of the factor set exceeds 300 dimensions.

Generally speaking, for a given number of training samples, the prediction ability of classification or regression model increases first and then decreases with the increase of the number of features. This is mainly because with the increase of the number (dimension) of features, the samples will become more sparse, so it is easier to find an ideal classification or regression method. But the increase of feature dimension will reduce the generalization ability of the model and prolong the training time of the model. Therefore, special methods need to be used to deal with high-dimensional features, that is, dimensionality reduction. At present, dimensionality reduction methods are mainly divided into two methods: feature selection and feature extraction. The difference between the two methods is whether to change the original feature space. For the quantitative stock selection model, although the factor dimension can improve the effectiveness of the stock selection model, it will also increase the training difficulty of the model, and some factors are seriously missing in the collected data, which will also affect the training of the model. Therefore, we deal with the feature selection of the stock selection factor set.

At present, there are two commonly used feature selection methods: variance based and information coefficient based. The methods based on variance include variance filtering and principal component analysis (PCA). The methods based on IC include the correlation calculation of different factors and the correlation calculation of factor and excess return. In this study, the method based on IC is used for factor selection. The factor selection process is shown in Algorithm 1.

As shown in Algorithm 1, the steps to get multifactor stock selection data set are as follows:

**Step 1 .**

*Factor Type Division*. According to the reference to previous literature results, we have divided the factors into categories, including valuation, growth, financial quality, debt repayment, profitability, and technical indicators.

**Step 2 .**

Manually screen the factors in the five categories, mainly to delete the factors with serious missing and repeated calculation methods.

**Step 3 .**

Calculate the correlation between factors and excess returns, and delete 50% of the factors with lower correlation.

**Step 4 .**

Calculate the correlation between factors and delete 50% of the factors with high correlation.

**Step 5 .**

Get the final quantitative stock selection data set.

In Step 2, we have excluded the factors with serious missing, but there will also be some missing values in the final quantitative stock selection factor set, which will affect the training and testing of the model. Therefore, we use the mean interpolation method for filling. However, some values cannot be completed by this method, such as PE. If the company is not profitable, PE is empty, which cannot be interpolated with the mean value, because if the mean value interpolation is adopted, it will be inconsistent with the actual situation. Therefore, in the experiment, we assign this kind of factor −1, so that after the data standardization, the value of this factor is also the smallest, and the impact on the experimental results will be very small.

In Step 3 and Step 4, the calculation of Spearman correlation coefficient is used to calculate the correlation, and the formula is shown as follows:

(1) $$\begin{array}{c} \text{Correl}\left(\text{X},\text{Y}\right)=\frac{\sum_{\text{i}=1}^{\text{n}}\left({\text{x}}_{\text{i}}-\bar{\text{X}}\right)\left({\text{y}}_{\text{i}}-\bar{\text{Y}}\right)}{\sqrt{\sum_{\text{i}=1}^{\text{n}}{\left({\text{x}}_{\text{i}}-\bar{\text{X}}\right)}^{2}{\left({\text{y}}_{\text{i}}-\bar{\text{Y}}\right)}^{2}}}. \end{array}$$

Finally, we constructed a multifactor stock selection data set containing 64 factors, as shown in Appendix A.

The factors involved in multifactor stock selection include financial statement data and stock market data. Since the financial statements of listed companies in China are published quarterly, the financial statement data we obtain are collected in quarterly units. Meanwhile, the stock market data can be collected in daily units. However, in order to reduce the cycle of stock selection, we use monthly data in our experiment. So, we need to unify the time granularity of different data.

Stock market data are mostly daily data. We can get the daily factors, such as daily yield, daily turnover, and daily closing price. Then, we convert the daily factors into monthly factors by summing, averaging, or calculating the standard deviation of the factor value of the current month.

We tried three methods to convert the quarterly financial data into monthly data.

### 2.1. Equal Difference Treatment

If the value of parameter *t* of stock A in the fourth quarter of year N−1 is *T*_*N*−1(season4)_ and the value of parameter *t* in the first quarter of year N is *T*_*N*(season1)_, then the value of parameter *t* in January of year N is as follows:

(2) $$\begin{array}{c} \left\{\begin{array}{c} T_{N\left(\text{January}\right)}=\frac{1}{2}\times T_{N\left(\text{season}1\right)}\times \frac{1}{3},T_{N\left(\text{season}1\right)}\geq T_{N-1\left(\text{season}4\right)},\\ T_{N\left(\text{January}\right)}=\frac{1}{2}\times T_{N\left(\text{season}1\right)},T_{N\left(\text{season}1\right)}<T_{N-1\left(\text{season}4\right)}. \end{array}\right. \end{array}$$

The value of parameter *t* in February is as follows:

(3) $$\begin{array}{c} T_{N\left(\text{February}\right)}=T_{N\left(\text{season}1\right)}\times \frac{1}{3}. \end{array}$$

The value of parameter *t* in March is as follows:

(4) $$\begin{array}{c} \left\{\begin{array}{c} T_{N\left(\text{March}\right)}=\frac{1}{2}\times T_{N\left(\text{season}1\right)},T_{N\left(\text{season}1\right)}\geq T_{N-1\left(\text{season}4\right)},\\ T_{N\left(\text{March}\right)}=\frac{1}{2}\times T_{N\left(\text{season}1\right)}\times \frac{1}{3},T_{N\left(\text{season}1\right)}<T_{N-1\left(\text{season}4\right)}. \end{array}\right. \end{array}$$

According to this method, the data in the financial statements of all listed companies from the first quarter of 2008 to the fourth quarter of 2020 are converted into the monthly financial statement data. The value of parameter *T* every month in any quarter is a simple linear relationship. If the value of parameter *t* in the quarter N is greater than (including equal) the value of the quarter N−1, the value of parameter *t* of each month in quarter N is an incremental arithmetic sequence. Conversely, if the value of parameter *t* in the quarter N is less than that in quarter N−1, the value of parameter *t* of each month in quarter N is a decreasing arithmetic sequence. It can simulate the trend of parameter *t* in each month in different quarters. However, due to the limitation of the granularity of data acquisition, this method may have some errors, which is different from the actual situation. Therefore, we propose the second processing method.

### 2.2. Equal Proportion Treatment

If the value of the parameter *t* of stock A in the first quarter of year N is *T*_*N*(season1)_ and the stock price of stock A at the end of each month in the first quarter of year *n* is *P*_*N*(January)_, *P*_*N*(February)_, and *P*_*N*(March)_, then the value of the parameter *t* in January, February, and March of year *n* is as follows:

(5) $$\begin{array}{c} \left\{\begin{array}{c} T_{N\left(\text{January}\right)}=T_{N\left(\text{season}1\right)}\times \frac{P_{N\left(\text{January}\right)}}{P_{N\left(\text{January}\right)}+P_{N\left(\text{February}\right)}+P_{N\left(\text{March}\right)}},\\ T_{N\left(\text{February}\right)}=T_{N\left(\text{season}1\right)}\times \frac{P_{N\left(\text{February}\right)}}{P_{N\left(\text{January}\right)}+P_{N\left(\text{February}\right)}+P_{N\left(\text{March}\right)}},\\ T_{N\left(\text{March}\right)}=T_{N\left(\text{season}1\right)}\times \frac{P_{N\left(\text{March}\right)}}{P_{N\left(\text{January}\right)}+P_{N\left(\text{February}\right)}+P_{N\left(\text{March}\right)}}. \end{array}\right. \end{array}$$

### 2.3. Shift Equal Proportion Treatment

Method 2 is to proportionate the stock price of this month to the parameters of this month, while the shift equal proportion is to proportionate the parameters of the current quarter by taking the stock price of each month of the previous quarter as the scale factor. This is because the release time of the financial report will be delayed compared with the stock price, that is, the financial statements of the first quarter will be released in April or May, which will affect the stock price of the second quarter instead of the current quarter.

If the value of the parameter *t* of stock A in the first quarter of year N is *T*_*N*(season1)_ and the stock price of stock A at the end of each month in the second quarter of year N is *P*_*N*(April)_, *P*_*N*(May)_, and *P*_*N*(June)_, then the value of the parameter *t* in April, May, and June of year *n* is as follows:

(6) $$\begin{array}{c} \left\{\begin{array}{c} T_{N\left(\text{April}\right)}=T_{N\left(\text{season}1\right)}\times \frac{P_{N\left(\text{April}\right)}}{P_{N\left(\text{April}\right)}+P_{N\left(\text{May}\right)}+P_{N\left(\text{June}\right)}},\\ T_{N\left(\text{May}\right)}=T_{N\left(\text{season}1\right)}\times \frac{P_{N\left(\text{May}\right)}}{P_{N\left(\text{April}\right)}+P_{N\left(\text{May}\right)}+P_{N\left(\text{June}\right)}},\\ T_{N\left(\text{June}\right)}=T_{N\left(\text{season}1\right)}\times \frac{P_{N\left(\text{June}\right)}}{P_{N\left(\text{April}\right)}+P_{N\left(\text{May}\right)}+P_{N\left(\text{June}\right)}}. \end{array}\right. \end{array}$$

We believe that the company's fundamental financial data can be reflected by the stock price, which is equivalent to linking the changes of factors with the changes of stock price. According to mapping the rise and fall of factor value with the rise and fall of stock price, the monthly factors are no longer strictly monotonous. Because the conclusion that the experiment needs to verify is that “the fluctuation law of stock price can be obtained through the calculation and analysis of multifactor”, method 2 and method 3 are reasonable. Although method 1 is the simplest, the changing trend of monthly factors generated by this method can only be increasing or decreasing in the quarter. In fact, neither it is necessarily strictly increasing or decreasing, nor it can reflect the changes of stock price. Therefore, method 1 is unreasonable.

The difference between method 2 and method 3 is the impact of the factors in the financial statements on the time stage of the stock price. Through experimental verification, the data sets obtained by method 2 and method 3 do not have much difference in the experimental performance, but method 2 can provide more samples. Therefore, we choose method 2 to convert the quarterly data into monthly data.

If the data scales differ greatly, the general method mainly optimizes the weight according to the error of large value. In order to avoid such errors, we scale different feature data to the same interval. There are two methods of feature scaling: normalization and standardization.

Normalization is to reduce the factor value in the data set to the [0, 1] interval and scale it with min-max:

(7) $$\begin{array}{c} X_{norm}^{\left(i\right)}=\frac{x^{\left(\text{i}\right)}-x_{\text{min}}}{x_{\text{max}}-x_{\text{min}}}, \end{array}$$

Standardization converts the factor value into a standard normal distribution with a mean value of 0 and a variance of 1:

(8) $$\begin{array}{c} X_{std}^{\left(i\right)}=\frac{x^{\left(\text{i}\right)}-\mu_{x}}{\sigma_{x}}, \end{array}$$

For most machine learning algorithms, the standardized method is easier to update the weight, so it is more practical. In the experiment, we use the standardized method to reduce the factor value to [−1, 1].

The stocks are classified into positive and negative cases according to the excess return. First, we sum the daily return of the stock in each month as the monthly total return of the stock. Second, we sum the daily return of the benchmark return (we choose the CSI 300 index as the benchmark return) as the monthly benchmark total return. The subtraction between the two is the monthly excess return. We think that it is the most intuitive performance of whether the stock can lead the market in a specified period of time and use an excess return to label stocks. The stock samples with positive excess return in the next month are marked as positive cases, and the stock samples with negative excess return in the next month are marked as negative cases. If the excess return of many stocks is close to 0, it indicates that these stocks are close to the market trend in the month and are not easy to be divided into positive or negative cases. The stocks close to 0 can be removed to make the positive and negative samples have greater differentiation (in the experiment, we select the first 40% of the samples as positive examples, the last 40% of the samples as negative examples, and eliminate the middle 20% of the samples).

## 3. Stock Selection Model Based on CNN

With the development of the financial market, a large number of data that may be related to stock are continuously generated. CNN has obvious advantages in processing high-dimensional data. Therefore, in order to make use of the characteristics of CNN in processing of two-dimensional data, we reorganize the multifactor data of individual stock into two-dimensional form and splice one-dimensional samples of the same stock at adjacent times to form a two-dimensional sample named “factor picture.” The length of the “factor picture” is the number of factors and the width of the “factor picture” is the number of spliced one-dimensional samples. Generally speaking, because data filtering leads to the discontinuity of samples in time, the longer the width, the fewer samples, because the more stringent the requirements. The “factor picture” is shown in Figure 1.

As shown in Figure 1, the “factor picture” is composed of 64 factors (EP, PB, ROE,…) and t−1 time spans factors of a stock. Rt is the relative rate of return at time *t*, which is used as the label. So, if there are 2000 stocks available in a time length, then we can get 2000 “factor picture” and their labels.

After the “factor pictures” are generated, these “factor pictures” are used as data sets to train and test the CNN model. The specific structure of the stock selection model based on CNN is shown in Figure 2.

In Figure 2, the time length of the factors is 3, and the constructed “factor picture” is a 63 × 3 two-dimensional picture. The process of the stock selection model based on CNN is shown in Algorithm 2.

As shown in Algorithm 2, we select the 2 × 2 convolution kernel W and perform the first convolution operation, as shown in the following equation:

(9) $$\begin{array}{c} \text{F}1_{t-2}=\left(PE_{t-3}*W1\right)+\left(PE_{t-2}*W2\right)+\left(PB_{t-3}*W3\right)+\left(PB_{t-2}*W4\right)+\text{bias,} \end{array}$$

where bias is the offset term.

Then, the input “factor picture” is convoluted in the horizontal and vertical directions to finally generate a 63 × 2 “first convolution result” with the 2 × 2 convolution kernel W. Then, the “first convolution result” is convoluted again with the 2 × 2 convolution kernel U, and a 62 × 1 “second convolution picture” is finally obtained.

Finally, we input the one-dimensional factor vector into the fully connected neural network and reconstruct the 63 × 1 vector as the input of the fully connected neural network. In order to improve the nonlinear fitting ability of CNN, we add ReLU activation function to the fully connected neural network and optimize the parameters according to the optimization method of the fully connected neural network.

We use two convolution layers in the model. Theoretically, more convolution layers can be added. However, due to the particularity of training data, all factors in this experiment have specific significance, which is different from the data mode of image processing, and the role of convolution layer is usually to make nonlinear combination between factors, Therefore, too many convolution layers do not have much significance. We compare the experimental results of one convolution layer and two convolution layers. The results show that the results of two convolution lays are better than the results of one convolution layer. We will not describe in detail here.

In the experiment, we did not use the pooling layer, which is the important part of CNN. Because the role of the pooling layer in CNN is to “blur” the convolution results and summarize the statistical features in the local region. In other words, the pooling layer can summarize the local features of the image region when only a small amount of information is lost, which is very useful for the dimensionality reduction and generalization of image recognition. However, in this experiment, as we said earlier, the factors constituting the “factor picture” are features with clear significance. If the pooling layer is used, some fine information of the factors will be lost, which will reduce the accuracy of the model.

In addition, combined with the basic principle of CNN, we believe that the factor arrangement order in the “factor picture” will have a certain impact on the training and prediction results. Different factor arrangement orders will affect the weight training in the convolution kernel. Even though the number of factors that we select is so big, there are too many possibilities for factor arrangement, which will be a very meaningful but heavy work. So, we will not focus on the different factor arrangements in this study. In the experiment, according to the type of factors, we put the factors of the same type in the adjacent position and then put the type factors that may interact in the adjacent position.

After completing the above work, the model is trained. We use the rolling training method if the data in time period [x, *x* + *n*] are selected as the training set and the data at time *x* + *n*+1 are used as the testing set. Rolling training not only ensures that each training set and testing set are adjacent at the time point but also ensures the number of testing results.

In the next part, we will introduce the experimental results of CNN stock selection model and compare them with the experimental results of decision tree, feedforward neural network, and support vector machine.

## 4. Experiment and Analysis

### 4.1. Experiment Design

In order to compare the effect of stock selection model based on CNN, we constructed stock selection models based on decision tree, SVM, and FNN, respectively, trained and tested different models under different parameters, obtained the optimal parameter set of each model, and then compared the model test effect under the optimal parameters.

We select 10 stocks by each stock selection models, buy on the first trading day of each natural month, and sell on the last trading day. In addition, we use CSI 300 index as the benchmark.

### 4.2. Evaluation Metrics

The test results are evaluated by annual return, sharp ratio, and max drawdown:

(10) $$\begin{array}{c} \text{annual return}=\text{total}\_\text{revenue}\times 12, \end{array}$$

where total_revenue is the total return of portfolio in a specified time period (month).

(11) $$\begin{array}{c} \text{sharpe ratio}=\frac{\text{excepted}\_\text{return}-R_{f}}{\text{std}\_\text{of}\_\text{portfolio}}, \end{array}$$

where excepted_return is the excepted rate of return of the portfolio; *R*_*f*_ is a constant representing the risk-free interest rate; std_of_portfolio is the standard deviation of the portfolio.

(12) $$\begin{array}{c} \text{max drawdown}=\max\frac{D_{i}-D_{j}}{D_{i}}\left(j>i\right), \end{array}$$

where *D*_*i*_ is the stock price on day *i*; *D*_*j*_ is the stock price on day *j*, and *j* > *i* means that day *j* is after day *i*.

### 4.3. Results and Discussions

#### 4.3.1. Stock Selection Model Based on Decision Tree

The parameters affecting the decision tree model include the height of the decision tree, the maximum number of leaf nodes, and the number of training sets. A too high decision tree may lead to overfitting in the division of some stock selection factors, but too low decision tree height will lead to underfitting. The restriction on the height of decision tree is the most direct means to control the complexity of decision tree model. When restricted, the algorithm will establish the optimal decision tree within the maximum number of leaf nodes, so it is also a means to prevent overfitting. It is related to the setting of decision tree height. Too many training sets may lead to internal conflicts in training data.

According to the experiment, we get the effect comparison of decision tree model under different parameter selection, as listed in Table 1.

As provided in Table 1, the effects under different parameters are quite different, which also explains the instability of the decision tree model. We get the best performance parameters of the decision tree model: the height of the decision tree is 25, the maximum number of leaf nodes is 50, and the number of training sets is 12. However, it can also be seen that limiting the super parameters can improve the performance of the model, but the instability of the decision tree can also be reflected; that is, the performance of different back-test indicators is inconsistent.

#### 4.3.2. Stock Selection Model Based on SVM

The parameters affecting the SVM model include the regularization coefficient C and the number of training sets. The larger the regularization coefficient C, the lower the tolerance for misclassification. On the contrary, the smaller the C, the higher the tolerance for misclassification. It is the key to control the “soft” and “hard” boundaries of SVM model. The value of C is related to the degree of overfitting. Too many training sets may lead to internal conflicts in training data.

According to the experiment, we get the effect comparison of SVM model under different parameter selection, as listed in Table 2.

As provided in Table 2, the results of SVM model are better than the results of decision tree model, but there are also unstable problems. We get the best performance parameters of support vector machine model: the regularization coefficient C is 1 and the number of training sets is 12.

#### 4.3.3. Stock Selection Model Based on FNN

The adjustment space of feedforward neural network model itself is more limited, and the main parameters include the number of hidden layers and the number of training sets.

According to the experiment, we have obtained the effect comparison of FNN model under different parameter selection, as listed in Table 3.

As listed in Table 3, the best performance parameters of FNN model are as follows: the number of hidden layers is 3 and the number of training sets is 12.

#### 4.3.4. Stock Selection Model Based on CNN

The parameters affecting the CNN model include learning rate, two-dimensional sample width, the number of convolution layers, the size of convolution kernel, and the number of training sets.

Through the experimental test, the lower learning rate can quickly converge to 100% training accuracy in the case of slightly higher model complexity. The performance is good enough. Improving the learning rate will make the final result easier to overfit. Therefore, in the model training, the learning rate is set to 0.0001. Because the samples to be processed by convolutional neural network must be organized into a two-dimensional form, that is, several monthly data are spliced together. This number determines the width of two-dimensional samples. Experiments show that too wide will lead to a too large time span of sample data, and the performance of financial factors in a longer time span is inconsistent. Therefore, the sample width is slightly smaller, which helps to ensure the consistency of internal data of the sample. On the other hand, if the width is too small, there is no room for convolution, so it has disadvantages. Because the training method adopted is rolling training, that is, continuously taking the two-dimensional sample data set of each month as the training set to supplement and improve the previous model, the number of data sets is not necessarily the more the better. For the same reason as the two-dimensional sample width, if the time span of the data set used is too large, the market laws learned by the model are also inconsistent. For example, if the data sets of all months from 2008 to 2018 are used as training sets, the effect of the model may not be good, because the internal laws of financial data are very complex and there are too many influencing factors. It is not possible to summarize the whole picture of financial data by several indicators. There are differences in market laws at different times and even at different times. It is better to choose data sets with a short span for training.

Through the above experimental results, we get the effect comparison of CNN model under different parameter selection, as listed in Table 4.

As provided in Table 4, the best performance parameters of CNN model are as follows: the sample width is 3, the number of training sets is 36, the number of convolution layers is 2, and the size of convolution kernel is 2 × 2.

Through the above experiments, we get the performance of four models when each model parameter is optimal, as listed in Table 5.

The experimental results of CNN and other comparison methods are listed in Table 5. It can be seen from the table that CNN obtains better results in the performance of annual return, sharp ratio, and max drawdown than all other comparison models. These improvements show that CNN is very suitable for stock selection in China's stock market. The comparison of annual return, sharp ratio, and max drawdown is shown in Figure 3.

Through the above comparison, we draw the following conclusions:

1. The stock selection model based on CNN has obvious advantages. The excess annual return and sharp ratio are the best among the four models. Although the sharp ratio of SVM model is close, the performance of SVM model in the max drawdown is very poor, and the excess annual return also has obvious disadvantages compared with CNN.
2. The stock selection model based on CNN is more stable. From the analysis of the effect of the single super parameter and the correspondence of the optimal model, the CNN is completely consistent, and the optimal model can be obtained by combining the optimal super parameters. The performance of SVM and decision tree model is very unstable, and there is a big gap between the super parameter value of the best model and the single super parameter analysis results.
3. The stock selection model based on CNN has stronger adaptability to the long-time training set. The effectiveness of the other three models decreases significantly with the increase of the scale of the training set. CNN performs better and better when the training data set is expanded. This also reflects that CNN has more advantages in processing data with time series.

## 5. Conclusion

Stock selection is an important strategy of quantitative trading. Good stock selection strategies can help get better returns. The existing studies have great problems in stock factor selection and stock selection. In order to solve these problems, we construct a multifactor stock selection data set based on the fundamental data and technical data of China's listed companies. We construct “factor pictures” by this data set as the input of the stock selection model based on CNN proposed in this study. We make full use of the advantages of CNN model in image classification. By constructing the “factor picture,” the effect of stock selection based on CNN can be significantly better than other models. Combined with certain financial knowledge, the data set can comprehensively cover all aspects of financial analysis on the premise of controllable factors and can better reflect the financial situation of companies, so as to establish a more accurate relationship between value and stock price. The experimental results show that the stock selection based on CNN can obtain better benefits in multifactor stock selection. The experimental results on China's stock market are carried out by constructing a dataset in a fixed market environment (China's stock market). In this article, we only construct the stock selection model through a single method, and there is no relevant research on the combination of multiple methods, such as the ensemble learning method represented by the decision tree. In the next step, we will mainly conduct relevant experimental research on the application of ensemble learning method in stock selection, so as to build a more complex stock selection model by integrating a variety of single methods, so as to improve the yield and stability of the model.

## Figures and Tables

**Figure 1:** Factor picture.

**Figure 2:** Stock selection model based on CNN.

**Figure 3:** The comparison of different stock selection methods.

**Algorithm 1:** Factor selection.

**Algorithm 2:** Stock selection model based on CNN.

**Table 1:** Results of decision tree under different parameters.

Training size	Leaf nodes	Depth	Benchmark	Annual return	Sharp ratio	Max drawdown
24	50	20	29864	15956	−0.0073	0.1946
36	50	20	45285	53892	0.02464	0.2008
48	50	20	35711	2871	0.0050	0.2199
24	50	25	29864	7042	−0.0027	0.2186
36	50	25	45285	57700	0.0236	0.2072
48	50	25	35711	33672	−0.0072	0.2689
24	50	30	29864	9193	−0.0083	0.1953
36	50	30	45285	44739	0.0168	0.2077
48	50	30	35711	5885	0.0078	0.2010
24	30	25	29864	43062	0.0059	0.2087
36	30	25	45285	35755	0.0145	0.2244
48	30	25	35711	5259	0.0051	0.2631
24	50	25	29864	10775	−0.0020	0.2065
36	50	25	45285	49842	0.0164	0.1878
48	50	25	35711	177	0.0092	0.2265
24	60	25	29864	2796	−0.0136	0.2071
36	60	25	45285	35754	0.0101	0.2066
48	60	25	35711	10825	0.0134	0.2355

**Table 2:** Results of SVM under different parameters.

Training size	Regular	Benchmark	Annual return	Sharp ratio	Max drawdown
	Coefficient				
24	1	29864	38751	−0.0152	0.2381
36	5	45285	35300	0.0150	0.2218
48	10	35711	34711	0.0236	0.2348
24	1	29864	38751	0.0144	0.2303
36	5	45285	−7198	−0.0060	0.2135
48	10	35711	−11128	−0.0056	0.2609
24	1	29864	19916	0.0082	0.2191
36	5	45285	2116	−0.0071	0.2188
48	10	35711	30951	0.0124	0.2273

**Table 3:** Results of FNN under different parameters.

Training size	Hidden layer	Benchmark	Annual return	Sharp ratio	Max drawdown
12	1	64367	5237	0.0023	0.2080
24	1	29864	1408	0.0192	0.2203
48	1	35711	11342	0.0043	0.2309
12	2	64367	32881	0.0472	0.2114
24	2	29864	4636	0.0150	0.2207
48	2	35711	27498	0.0236	0.2348
12	3	64367	38002	0.0352	0.2114
24	3	29864	26367	0.0250	0.1913
48	3	35711	29701	0.0236	0.1967

**Table 4:** Results of CNN under different parameters.

Training size	Sample width	Type	Benchmark	Annual return	Sharp ratio	Max drawdown
36	3	1	45285	64351	0.0146	0.2176
36	3	2	45285	61248	0.0196	0.2420
36	3	3	45285	20171	0.0134	0.2188
24	3	1	29864	12915	−0.0011	0.2437
24	3	2	29864	75060	0.0243	0.2225
24	3	3	29864	15195	−0.0135	0.2548
36	6	1	45285	6464	−0.0003	0.2171
36	6	2	45285	27737	0.0159	0.2060
36	6	3	45285	58898	0.0194	0.2041
24	6	1	29864	−6565	−0.0038	0.2429
24	6	2	29864	−24867	−0.0210	0.2394
24	6	3	29864	12791	−0.0013	0.2159

**Table 5:** Best performance of four models.

Model	Benchmark	Annual return	Sharpe ratio	Max drawdown
Decision tree	45285	64267	0.0506	0.1929
SVM	45285	66376	0.0619	0.2326
FNN	45285	38001	0.0335	0.2114
CNN	45285	71248	0.0696	0.2150

**Table 6:** The Stock Selection factors.

No.	Factor	Type of factor	Description
1	TMV	Value	Total market value
2	CPs	Value	The average daily closing price of individual stocks in the last month is taken as logarithm
3	EPS	Value	Earnings per share
4	TOIS	Value	Total operating income per share
5	PE	Value	Price-to-earnings ratio, PE = total market value/net profit = PRICE/EPS
6	PECut	Value	Price-to-earnings cut ratio, PECut = total market value/net profit after deducting nonrecurring profit and loss
7	PB	Value	Price-to-book ratio, PB = total market value/net assets = = PRICE/BPS
			BPS : BOOK PER SHARE
8	PS	Value	Price-to-sales ratio, PS = total market value/operating income = PRICE/SPS
			SPS : SALE PER SHARE
9	PNFC	Value	Price-to-net cash flow, PNFC = total market value/net cash flow
10	POCF	Value	Price-to-operating cash flow, POCF = total market value/operating cash flow
11	ORYY	Growth ability	Year-to-year growth rate of operating revenue
12	NPYY	Growth ability	Year-to-year growth rate of net profit
13	OCFYY	Growth ability	Year-to-year growth rate of operating cash flow
14	ROEYY	Growth ability	Year-to-year growth rate of ROE
15	ROE	Financial quality	Return on equity, ROE = net profit/net assets
16	ROA	Financial quality	Return on assets, ROA = [net income + interest *∗* (1−tax rate)]/total assets
17	GPM	Financial quality	Gross profit margin, GPM = gross profit/operating income *∗* 100%
18	NPM	Financial quality	Net profit margin, NPM = net profit/operating income *∗* 100%
19	AT	Financial quality	Asset turnover, AT = total revenue/total asset
20	RTR	Financial quality	Receivables turnover ratio
21	CAT	Financial quality	Current assets turnover
22	IT	Financial quality	Inventory turnover
23	FAT	Financial quality	Fixed assets turnover
24	TANA	Debt-paying ability	TANA = total assets/net assets
25	NCLNA	Debt-paying ability	NCLNA = noncurrent liabilities/net assets
26	Cash ratio	Debt-paying ability	Cash ratio = (cash + cash equivalents)/current liabilities *∗* 100%
27	Current ratio	Debt-paying ability	Current ratio = current assets/current liabilities
28	Quick ratio	Debt-paying ability	Quick ratio = liquid capital/current liabilities
29	Equity ratio	Debt-paying ability	Equity ratio = total liabilities/total owners' equity
30–33	AANm	Profitability	The arithmetic average value of the daily turnover rate multiplied by the daily yield of individual stocks in the last N months, *N* = 1, 3, 6, and 12
34–37	SDNm	Profitability	Standard deviation of daily return series of individual stocks in the last N months, *N* = 1, 3, 6, and 12
38–41	ARNm	Profitability	Average value of daily return series of individual stocks in the last N months, *N* = 1, 3, 6, and 12
42–45	AT_Nm	Profitability	Average value of daily turnover rate series of individual stocks in the last N months, *N* = 1, 3, 6, and 12
46	RSC	Profitability	Ratio of sales to cost, RSC = cost of sales/net sales *∗* 100%
47	DAR	Profitability	Debt asset ratio, DAR = total indebtedness/total assets *∗* 100%
48	EBIT	Profitability	Earnings before interest and tax, EBIT = net profit + income tax + interest
49	ROA_Y	Profitability	Return on assets in one year
50	ROIC_Y	Profitability	Return on invested capital in one year, ROIC = (net income − tax)/total capital *∗* 100%
51	EPSYY	Profitability	Year-to-year growth rate of EPS
52	NCFYY	Profitability	Year-to-year growth rate of net cash flow from operating activities per share
53	SPYY	Profitability	Year-to-year growth rate of sales profit
54	NPYY	Profitability	Year-to-year growth rate of net profit attributable to shareholders of the parent company
55	NATY	Profitability	Growth rate of net assets per share relative to the beginning of the year
56	TATY	Profitability	Growth rate of total assets relative to the beginning of the yea
57	TORYY	Profitability	Year-to-year growth rate of total operating revenue
58	TORYYS	Profitability	Year-to-year growth rate of total operating revenue in single quarter
59	OPYYS	Profitability	Year-to-year growth rate of operating profit in single quarter
60	NPYYS	Profitability	Year-to-year growth rate of net profit attributable to shareholders of the parent company in single quarter
61	MACD	Technical indicators	Moving average convergence divergence
62	RSI	Technical indicators	Relative strength index
63	PSY	Technical indicators	Psychological line
64	BIAS	Technical indicators	

We constructed a multi-factor stock selection data set containing 64 factors by the method based on Information Coefficient.

## Data Availability

The data used to support the findings of this study are available from the corresponding author (e-mail lipengfei@ucas.ac.cn) upon request.
